The article "Analysis of the role and robustness of artificial intelligence in commodity image recognition under deep learning neural network" was retracted in 2024. Reasons: duplicate publication; overlap with earlier publications; compromised peer review; unreliable results or conclusions.

# Analysis of the role and robustness of artificial intelligence in commodity image recognition under deep learning neural network

**DOI:** 10.1371/journal.pone.0235783

**Published:** 2020-07-07

**Authors:** Rui Chen, Meiling Wang, Yi Lai

**Affiliations:** School of Communications and Information Engineering, Xi’an University of Posts and Telecommunications, Xi’an, China; University College London, UNITED KINGDOM

## Abstract

In order to explore the application of the image recognition model based on multi-stage convolutional neural network (MS-CNN) in the deep learning neural network in the intelligent recognition of commodity images and the recognition performance of the method, in the study, the features of color, shape, and texture of commodity images are first analyzed, and the basic structure of deep convolutional neural network (CNN) model is analyzed. Then, 50,000 pictures containing different commodities are constructed to verify the recognition effect of the model. Finally, the MS-CNN model is taken as the research object for improvement to explore the influence of label errors (p = 0.03, 0.05, 0.07, 0.09, 0.12) with different parameter settings and different probabilities (size of convolutional kernel, Dropout rate) on the recognition accuracy of MS-CNN model, at the same time, a CIR system platform based on MS-CNN model is built, and the recognition performance of salt and pepper noise images with different SNR (0, 0.03, 0.05, 0.07, 0.1) was compared, then the performance of the algorithm in the actual image recognition test was compared. The results show that the recognition accuracy is the highest (97.8%) when the convolution kernel size in the MS-CNN model is 2*2 and 3*3, and the average recognition accuracy is the highest (97.8%) when the dropout rate is 0.1; when the error probability of picture label is 12%, the recognition accuracy of the model constructed in this study is above 96%. Finally, the commodity image database constructed in this study is used to identify and verify the model. The recognition accuracy of the algorithm in this study is significantly higher than that of the Minitch stochastic gradient descent algorithm under different SNR conditions, and the recognition accuracy is the highest when SNR = 0 (99.3%). The test results show that the model proposed in this study has good recognition effect in the identification of commodity images in scenes of local occlusion, different perspectives, different backgrounds, and different light intensity, and the recognition accuracy is 97.1%. To sum up, the CIR platform based on MS-CNN model constructed in this study has high recognition accuracy and robustness, which can lay a foundation for the realization of subsequent intelligent commodity recognition technology.

The article "Analysis of the role and robustness of artificial intelligence in commodity image recognition under deep learning neural network" was retracted in 2024. Reasons: duplicate publication; overlap with earlier publications; compromised peer review; unreliable results or conclusions.

## 1. Introduction

Nowadays, large shopping malls, supermarkets, and small retail stores offer a wide variety of goods for consumers to choose, which brings rich and convenient shopping experience to people and greatly stimulates and promotes the speed of social development. At present, the operation mode often adopted in the retail market is storekeeper self-operation, consumer self-selection, single duty, and long hours business, and convenience stores can bring convenient and timely shopping experience to consumers and improve the efficiency of life services [1]. At the beginning, barcode technology was mainly used to identify commodities. It needs to identify each commodity with barcode printed on the outer packaging. However, the printed bar codes of different commodities are not the same, so it is necessary to find the location of bar codes manually to assist machine recognition, so the degree of automation is relatively low [2,3]. In recent years, automated retail stores have appeared successively at home and abroad. This store uses artificial intelligence technology to realize automated and unmanned sales of goods. In order to liberate productivity, it is very important to use image vision technology to identify goods.

The ideal commodity recognition technology is to complete the recognition only through computer equipment and image acquisition equipment, and the intelligent recognition of commodity image requires high recognition accuracy, high recognition speed, and high degree of automation. When identifying and classifying goods based on the image recognition technology, the main technology is machine learning algorithm. At present, deep learning algorithms are most widely used in the field of computer vision [4]. Too et al. (2019) constructed a blade image recognition system based on deep convolutional neural network, and the results show that the recognition accuracy of this method is up to 99.75% [5]. Compared with other classical models, MS-CNN model in deep learning has the characteristics of fast convergence, low error detection rate, and high recognition accuracy. Dai et al. (2017) proposed a method for fundus image lesion recognition based on MS-CNN model, and found that the recognition accuracy of this method was 99.7% and the recall rate was 87.8% [6]. Zhai et al. (2019) showed that data training in MS-CNN model could improve the extraction effect of robust features and avoid the occurrence of overfitting [7]. Therefore, in order to meet the demand of automatic recognition of commodities, and to improve the recognition efficiency and save costs, I conducted the research on intelligent CIR technology based on deep learning algorithm to meet the application demand of automatic recognition of individual merchants.

The article "Analysis of the role and robustness of artificial intelligence in commodity image recognition under deep learning neural network" was retracted in 2024. Reasons: duplicate publication; overlap with earlier publications; compromised peer review; unreliable results or conclusions.

## 2. Literature review

### 2.1. Research progress of commodity image recognition technology

Among the automated commodity recognition technologies, bar code recognition technology is the most mature. Ren et al. (2018) found that the index number of barcodes can accelerate the detection speed, and the application of DNA barcode in biometrics can effectively realize the recognition of different species [8]. Lin et al. (2017) found that automatic location of bar codes is a key step in the bar code image recognition system, while the generalization of traditional bar code location algorithm is extremely limited, so a method for accurate location of bar codes is proposed, which can effectively realize the recognition of bar codes in any region [9]. However, the barcode will be damaged in the process of commodity transportation, which will affect the effect of barcode recognition. Then people introduced the wireless radio frequency recognition technology (RFID), which is used widely. Zou et al. (2017) applied COTS RFID technology to gesture recognition, and finally found that the recognition accuracy in different positions was above 90% with strong anti-interference [10]. Cappai et al. (2018) combined RFID technology with DNA molecular technology and applied it to the recognition of meat commodities. Finally, they found that it can realize intelligent recognition of commodities in a short time and greatly save costs [11]. With the rapid development of computer vision technology, the research on the application of vision technology in commodity recognition has also received great attention, among which SIFT/SURF feature point recognition technology is the most classic. Hou and Zhou (2017) selected the multi-feature scale of key points based on Gabor kernel function and applied it to image recognition, and finally found that it could improve the reliability of image feature matching [12]. Liu et al. (2018) proposed a recognition method for local texture and structure features based on SIFT and HOG, and finally found that the method proposed in this study has higher performance [13]. It shows that SIFT and other methods can improve the accuracy and speed of image recognition, but SIFT and SURF technologies are all used to extract local feature points of images, and the accuracy of extracting local feature points in mass image recognition is relatively low.

### 2.2. Application of deep learning in image recognition

There are more and more researches on the application of deep learning in image recognition, and a lot of studies show that the image recognition algorithm based on deep learning can effectively improve the accuracy of recognition. Bychkov et al. (2018) proposed a model for cancer image recognition and prediction based on deep network [14]. Wurfl et al. (2018) proposed an image reconstruction method based on the deep learning framework, and finally found that its peak signal to noise ratio increased by 23%, and the network model could complete automatic learning [15]. Wang et al. (2019) proposed a method for fuzzy image recognition based on deep convolutional neural network, and found that this method has higher performance than Alexent and GoogleNet [16]. Zhu et al. (2019) proposed a vehicle image feature recognition method based on deep learning and applied it to VeRi and VehicleID databases for verification, and found that this method has a high recognition performance for vehicle image recognition [17]. Based on deep learning, Nodera et al. (2019) proposed a method for patient resting needle electromyography image recognition and classification, and it was found that the method could effectively complete signal classification [18]. Barbedo (2019) proposed a method for disease recognition in plant images based on deep learning, and the results showed that the average recognition accuracy of this method was 15% higher than the original image [19].

The article "Analysis of the role and robustness of artificial intelligence in commodity image recognition under deep learning neural network" was retracted in 2024. Reasons: duplicate publication; overlap with earlier publications; compromised peer review; unreliable results or conclusions.

To sum up, deep learning algorithms are widely used in image recognition and can achieve high detection results. However, there are few studies on its application in CIR. Therefore, an algorithm for CIR based on DLNN model is proposed, and through the construction of the commodity image database, the training and verification of the model is carried out, then the recognition accuracy and robustness of the model is analyzed. The purpose of this study is to provide theoretical basis for the research of intelligent commodity recognition system.

## 3. Methodology

### 3.1. The characteristics of commodity images

In order to increase consumers’ desire to buy commodities and ensure that the commodities are highly recognizable, manufacturers tend to diversify their packaging designs. The design of color, shape, and character style of commodity package makes commodities have rich image features. Among them, the commodity packaging has rich and bright colors, which can cause a strong visual impact to consumers. The color space is mainly divided into two categories: digital image processing and hardware analysis for monitors. The most commonly used spaces of the two types of color space are red-green-blue (RGB) space and hue-saturation-value (HSV) space [20]. The color distribution of these two spaces is shown in Fig 1.

The article "Analysis of the role and robustness of artificial intelligence in commodity image recognition under deep learning neural network" was retracted in 2024. Reasons: duplicate publication; overlap with earlier publications; compromised peer review; unreliable results or conclusions.

**Fig 1:** Color distribution RGB space and HSV space (A is RGB space; B is HSV space).

It can be concluded from Fig 1A that all the studies in RGB space are composed of red, green, and blue. There are 255 levels in each channel, and the channel value is any value in 0–255. The total color can be obtained by adding the three channel vectors, and the calculation equation is as follows.

$$\vec{T}=\vec{R}+\vec{G}+\vec{B}$$ (1)

It can be concluded from Fig 1B that the dominant color of HSV space is Hue, and the different Hue values are represented by the cone Angle (0–360°), where red is 0°. Gray histogram is a way to count the number of pixels in the image pixel value. It can normalize the image and then obtain the ratio between the number of pixels in each image and the total number of pixels in the image.

In addition to the color, the shape of the outer package is also different for different types of goods. For example, the packaging of drinks is usually canned and bottled, snacks are packaged in bags, yogurt commodities are packaged in boxes, and so on. In the process of digital image processing, the shape features of commodity images can be divided into regional features and feature boundary features. The main methods used to describe the regional characteristic shape include area, concave and convex type, horizontal and vertical ratio and so on. The main methods used to describe the shape of feature boundary include Fourier shape descriptor and Hough transform detection [21]. Taking the bottled beverage as an example, its characteristic outline is described. The effect is shown in Fig 2. In contour diagram of Fig 2B, the blue closed curve is composed of countless points on the contour boundary of the commodity, while the red line is the direction of the commodity in the closed curve, and the green circle is the center of gravity in this area.

**Fig 2:** Commodity original and outline images (A is the original image; B is the outline image).

The texture feature of commodity image is a relatively complicated feature. From the perspective of vision, the local texture of the image often shows the irregular state, but the overall image shows the regularity and periodicity. Methods commonly used to filter texture and edge features in images include Sobel, Prewitt, and Canny, etc. Taking COINS as an example, the detection effect of different edge detectors is shown in Fig 3.

**Fig 3:** Results of different edge detectors (A is the original image; B is the Sobel detector; C is the Prewitt detector; D is Canny detector).

Point feature refers to the key points in the image. By analyzing the image with these local key feature points, the image can be accurately positioned and the accuracy of image recognition can be improved. The feature points of Scale independent feature transform (SIFT) mainly adopt the local maximum value of image and scale space [22]. The method adopted by Speeded up robust feature (SURF) is like that of SIFT, but it mainly uses gaussian filter to response [23], so the computation efficiency is higher.

The article "Analysis of the role and robustness of artificial intelligence in commodity image recognition under deep learning neural network" was retracted in 2024. Reasons: duplicate publication; overlap with earlier publications; compromised peer review; unreliable results or conclusions.

### 3.2. DLNN

Machine learning is a way of exploring computer simulations and realizing human learning behavior. New knowledge and skills are obtained to reorganize existing knowledge structures and improve its own performance. As a further derivative of machine learning, deep learning has more intelligent characteristics. CNN is the first learning algorithm to successfully train the multi-layer network structure, which can use spatial relationship to reduce the number of learning parameters and improve the training performance of forward BP algorithm. The CNN model is a multi-layer artificial neural network, in which each layer is composed of multiple two-dimensional planes, and each plane is composed of multiple independent neurons. The structure diagram of CNN is shown in Fig 4.

**Fig 4:** Schematic diagram of CNN.

The initialization of the CNN model is mainly to initialize the convolution kernel and bias in the convolutional layer and output layer. The convolution kernel (weight) is often treated with random initialization, while the bias is usually 0. When the forward propagation of the CNN model is calculated, the input layer, convolutional layer, pooling layer (sampling layer), and output layer of the structure are calculated in different ways. There is no exact input value in the input layer, only one output vector value, that is, the picture size matrix of 32*32; the input value of the convolutional layer comes from the input layer or pooling layer, and the feature graphs in the convolutional layer all have a convolution kernel of the same size. Different convolutional kernel sizes have an important influence on the convergence speed and recognition accuracy of the CNN model. Assuming the size of the convolution kernel is 2*2, the size of the input feature graph is 4*4, then the size of the output feature graph of the convolutional layer is 3*3. There are 6*12 convolution kernels in the SC3 layer in Fig 5, so the different feature graphs in the convolution layer are all different convolution kernels to carry out convolution in the feature graph of the upper layer. After accumulation, bias is obtained, and Sigmod function is used for calculation. The pooling layer mainly carries on the sampling processing to the characteristic graph output of the upper layer, that is, the aggregate statistics is carried out on the adjacent small regions of the characteristic graph of the upper layer.

The article "Analysis of the role and robustness of artificial intelligence in commodity image recognition under deep learning neural network" was retracted in 2024. Reasons: duplicate publication; overlap with earlier publications; compromised peer review; unreliable results or conclusions.

**Fig 5:** The construction process of CIR platform.

The calculation process of reverse weight adjustment is the most complicated process in the CNN model. The residual of the output layer of CNN model is calculated differently from that of the middle layer, while the residual value of the output layer is the error value of the output value and class standard value. The calculation equation of the residual value of the output layer is as follows.

$$\begin{array}{ll} \delta_{i}^{\left(n_{1}\right)}= & \frac{\partial }{\partial z_{i}^{\left(n_{1}\right)}}\frac{1}{2}{\left\|y-h_{W,b}\left(x\right)\right\|}^{2}\\ & =-\left(y-a^{\left(n_{1}\right)}\right)\cdot f^{\prime }\left(z^{\left(n_{1}\right)}\right) \end{array}$$ (2)

In Eq 2, n_1_ is the output layer, y is the output value, and h_W,b_ is the class value, a is the constant calculated after the equation is deformed.

If the next layer of the convolution layer is the pooling layer, then the residual of the pooling layer is extended by the Kronecker commodity with the Scale*Scale full 1 matrix. Furthermore, the residual dimension of pooling layer is consistent with the dimension of the previous output characteristic graph, and the residual is obtained by convolution calculation. If the next layer below the pooling layer is the convolutional layer, then the convolutional kernel needs to be rotated by 180°, and the volume and proof are extended to 0 to find the unit associated with the weight in the feature graph. Finally, the convolution kernel is used to process convolution and the residual of pooling layer is obtained.

In the CNN model, the Softmax layer is mainly used as the output layer. Assuming the number of samples in the sample set is m, then the sample set is expressed as {(*x*^1^, *y*^1^), (*x*^2^, *y*^2^), ⋯,(*x*^*m*^, *y*^*m*^)}. Among them, x is the vector value of the input sample, y is the category label of the sample, and *y* ∈ {1, 2, ⋯, k}. Supposing the input value of the Softmax layer is z, then the output value is Z = f(z). Among them, Z is the vector m dimensional column. At this point, the expression of the Softmax classifier is as follows.

$$Z=f\left(z^{j}\right)=\frac{\text{exp}\left(z^{j}\right)}{\sum_{j=1}^{k}\text{exp}\left(z^{j}\right)}$$ (3)

Then the normalized expression is as follows.

$$p\left(y=j|x\right)=f\left(z^{j}\right)=\frac{\text{exp}\left(z^{j}\right)}{\sum_{j=1}^{k}\text{exp}\left(z^{j}\right)}$$ (4)

The sum of the probabilities between the sample sizes is 1. The loss function is applicable to measure the difference between the label value of the input sample predicted by the neural network and the actual value, then the function can be denoted as L(θ). Among them, θ is the current neural network space. Softmaxloss function is used in the CNN model of this study, and its expression is as follows.

$$L\left(\theta \right)=-\text{log}\left[f\left(z^{m}\right)\right]=-\text{log}\left[\frac{\text{exp}\left(z^{m}\right)}{\sum_{j=1}^{k}\text{exp}\left(z^{m}\right)}\right]$$ (5)

In Eq 5, m is the true label value. The larger the value of z^m^ is, the smaller the value of L(θ) is. When f(z^m^) approaches 1, L(θ) approaches 0; while when f(z^m^) approaches 0, L(θ) approaches infinity.

The article "Analysis of the role and robustness of artificial intelligence in commodity image recognition under deep learning neural network" was retracted in 2024. Reasons: duplicate publication; overlap with earlier publications; compromised peer review; unreliable results or conclusions.

After calculating residuals of different layers in the CNN model, the weight value and bias in the network are adjusted and updated, and the performance of the network is adjusted through repeated training.

### 3.3. Construction of CIR platform

In this study, 80 kinds of popular drinks, snacks, daily necessities, and other commodities in supermarkets are selected as the objects of the CIR experiment. According to the appearance characteristics of different commodities, the experimental platform for commodity images is built, including the collection, preprocessing, database generation, and expansion of commodity images. The specific experimental process is shown in Fig 5.

In this study, CMOS camera is used to shoot commodity images, with a resolution of 640*480 pixels. Then the ordinary LED lamp is selected as the shooting light source, and the illumination mode is diffuse. Then, VS013 and Python IDLE are selected as the main development environment, OpenCV, the open source database of computer vision, is used as the image processing tool, and MXNet is used as the experimental framework of deep learning. The process of this experiment is completed in Windows system.

Then, the commodity image is collected. Cuboid commodities are mainly shot on 6 planes, and 10 images are shot on each plane. Cylindrical goods are mainly shot by rotating the plane, and 8 images are shot for each rotation of 60°. Plastic packaging commodities are mainly photographed in front and back 2 planes, and 20 images are shot for each plane. The length and width of all images captured in this experiment are set to 350*350 mm, and the original size of commodity images in the CNN model is 640*480, all of which are RGB space colors. Then, the commodity image is preprocessed, and the target threshold is determined by OTSU, and the image is segmented by threshold. First, the color image obtained by shooting is converted to the gray image, then the calculation equation of the gray value is as follows.

The article "Analysis of the role and robustness of artificial intelligence in commodity image recognition under deep learning neural network" was retracted in 2024. Reasons: duplicate publication; overlap with earlier publications; compromised peer review; unreliable results or conclusions.

Gary=R⋅0.299+G⋅0.587+B⋅0.114 (6)

Then the OTSU is used to segment the image. By marking the pixels in the contour of the image, the contour area of the target commodity is determined, and the edge information of the commodity image is obtained and the region of interest (ROI) is extracted. The processed image size is 300*300, and pepper, salt, and gaussian noise are added to the commodity image, and the image rotation from different angles is processed to improve the accuracy of the model training.

### 3.4. CIR based on DLNN

The classic CNN is Lenet-5 network, and the input sample size is usually 28*28, which can’t be used for the recognition of complex category images. However, commodity images have more complexity. Therefore, the MS-CNN model is taken as the research object. Meanwhile, in order to improve the learning efficiency of the network, the MS-CNN model is improved. The main improvement steps are as follows: I. the size of the input sample is increased; II. the activation function in the network is improved. The gradient value of tanh() function in the original network is small. Therefore, when the input sample size is large, the training time will be too long. Therefore, the linear coefficient α is increased based on the original function, α = 0.16; III. the number of neurons in the output layer is adjusted; IV. the depth of hidden layer is increased; V. network is trained based on Dropout training idea. Therefore, the MS-CNN model framework constructed in this study is shown in Fig 6.

**Fig 6:** The structure diagram of the modified MS-CNN model.

The specific parameters set in the MS-CNN model used in this study are shown in Table 1.

**Table 1:** Parameters of all layers in MS-CNN model.

MS-CNN model	Number of feature images	Size of feature images	Trainable parameters	The connection point	Other parameters
The input layer		46*46			
Convolution layer 1	10	40*40	500	800000	Convolutional kernel 3*3/10
Pooling layer 1	10	20*20	100	20000	
Convolution layer 2	20	16*16	520	133120	Convolutional kernel 5*5/20
Pooling layer 2	20	8*8	100	6400	
Convolution layer 3	60	4*4	1560	24960	Convolutional kernel 5*5/50
Pooling layer 3	60	2*2	120	1200	
The fully connected layer		2*2			
The output layer					Neuron 40

The maximum number of iterations set in this study is 4500, and the error value will be output once every 10 times. Then different types of commodity pictures are selected from Baidu photo library to build the detection database. In the end, a total of 50,000 pictures containing different commodities are included to verify the recognition effect of the model constructed in this study.

## 4. Results and discussion

### 4.1. Effects of different parameter settings on the recognition accuracy of MS-CNN model

In order to evaluate the effect of convolution kernel size and Dropout rate on the recognition accuracy of MS-CNN model, in this study, MS-CNN model is trained using the self-constructed commodity image database. Firstly, the training method in the MS-CNN model is set as SGD method, and the Dropout discard rate is 0.1. Then, the influence of the size change of convolution kernel on the recognition accuracy is compared. It can be concluded from Fig 7A that different convolution kernel sizes have little influence on the accuracy and robustness of CIR. When the training method in the MS-CNN model is SGD method and the convolution kernel size in convolutional layer 1 is 3*3, the influence of Dropout discard rate change on recognition accuracy is compared. As concluded from Fig 7B, Dropout rate has a great influence on the accuracy and robustness of commodity recognition [24]. When Dropout rate is 0.6, the loss value is the largest, when Dropout rate is 0.1, the loss value is the smallest.

The article "Analysis of the role and robustness of artificial intelligence in commodity image recognition under deep learning neural network" was retracted in 2024. Reasons: duplicate publication; overlap with earlier publications; compromised peer review; unreliable results or conclusions.

**Fig 7:** The influence of different parameters on the recognition accuracy of MS-CNN model (A is the change of convolution kernel size; B is the change of Dropout rate).

Then, the training results of MS-CNN model with different parameters are compared. It can be concluded from Table 2 that the average recognition accuracy is the highest (97.8%) when the size of the convolution kernel is 2*2 and 3*3, the training time is the shortest (340s) when the size of the convolution kernel is 2*2, and the training time is the longest when the convolution kernel size is 10*10 (1003s). The average recognition accuracy is the highest (97.8%) when the Dropout rate is 0.1. The training time is the shortest (340s) when Dropout rate is 0.6, but the recognition accuracy is the lowest (82.5%). It is found that with the increase of convolution kernel size, the accuracy rate of MS-CNN model in CIR is more than 96%, but the training time increases. This may be because too large convolution kernel size will increase the computation amount of network operation, thus increasing the training time [25]. The size of the convolution kernel is 2*2. If the size of the convolution kernel is too small, the output image information will be too little and the features in the image will be too bad. The large size of the convolution kernel will lead to the increase of calculation quantity, which is not only bad for the increase of model depth, but also reduces the performance of model calculation [26]. While the convolution kernel of size 3*3 is widely used in various models. In order to ensure the recognition accuracy and operation efficiency of the network, the convolutional kernel with sizes of 3*3 and 5*5 and parameters with Dropout rate of 0.1 are finally selected for subsequent experiments.

The article "Analysis of the role and robustness of artificial intelligence in commodity image recognition under deep learning neural network" was retracted in 2024. Reasons: duplicate publication; overlap with earlier publications; compromised peer review; unreliable results or conclusions.

**Table 2:** The influence of different parameters on the recognition efficiency of MS-CNN model.

Parameters	Changes	The average accuracy rate	Training time (s/times)
Convolution kernal size	2*2	97.8%	340
	3*3	97.8%	341
	5*5	97.4%	413
	7*7	97.4%	626
	9*9	97.5%	802
	10*10	96.1%	1003
Dropout rate	0.1	97.8%	341
	0.2	97.7%	342
	0.3	97.2%	342
	0.4	96.0%	345
	0.5	91.4%	359
	0.6	82.5%	340

### 4.2. Effect of label modification on prediction accuracy of MS-CNN model

According to the test results, the initial learning rate is set as 0.01, the training method is set as stochastic gradient descent (SGD), the size of the initial convolution kernel is set as 3*3, the Dropout rate is set as 0.1, and the maximum number of iterations is set as 10000 to conduct the CIR experiment. Then, the p value of label modification probability is randomly selected within the range of the commodity image, and the difference of prediction accuracy under different probabilities is first compared. As concluded from Fig 8A, as the value of p increases, the accuracy of network prediction declines sharply when labels are wrong. The error is the largest when the p value is 0.12. As concluded from Fig 8B, with the increase of p value, the difference between the accuracy value of the final prediction of this research model and the accuracy value of the prediction without errors also increases. When p is 0.03 and 0.05, the difference between the predicted accuracy values is small.

**Fig 8:** The influence of label modification on the prediction accuracy of MS-CNN model (A is the change of the final prediction accuracy value of the model in this study; B is the change in the final prediction accuracy value when the label is wrong).

As concluded from Table 3, when the p value increases to 0.09 and 0.12, the accuracy of network prediction will decline to a very low level; however, the prediction accuracy of MS-CNN model constructed in this study can reach 96% when the p value is 0.12; the prediction accuracy drops by only 3.3% compared with the prediction accuracy when the labels are correct, which indicates that the MS-CNN model constructed in this study effectively reduces the negative impact of commodity image labeling errors and effectively improves the robustness of CIR, which is consistent with the research results of Xuan et al. (2017) [27].

**Table 3:** Comparison of prediction accuracy of different algorithms.

P-value	Accuracy_orig	Accuracy_modify	Accuracy_error
0.03	0.993	0.982	0.901
0.05	0.993	0.975	0.869
0.07	0.993	0.967	0.326
0.09	0.993	0.965	0.197
0.12	0.993	0.960	0.155

Accuracy_orig represents the accuracy of MS-CNN prediction when no errors are marked; Accuracy_modify represents the prediction accuracy of this research model when marking errors; Accuracy_error is the accuracy of MS-CNN prediction when marked wrong.

The article "Analysis of the role and robustness of artificial intelligence in commodity image recognition under deep learning neural network" was retracted in 2024. Reasons: duplicate publication; overlap with earlier publications; compromised peer review; unreliable results or conclusions.

### 4.3. MS-CNN module for detection of CIR

In order to test the effect of building MS-CNN model in CIR in this study, several commodity databases generated in the early stage are used to verify the recognition effect of MS-CNN model. In order to test the robustness of the algorithm proposed in this study, salt and pepper noise is introduced in the model training. The process of adding noise is as follows. I. SNR in the range of [0,1] is selected. II. the total number of pixels in the training image is calculated, and (1-SNR)/ total number of pixels noise points is calculated. III. a pixel in the training image is randomly selected and the pixel value of the position is set to 0 or 255. IV. the previous step is repeated until the image is saved. In the process of the experiment, the SNR values of 0, 0.03, 0.05, 0.07 and 0.1 are selected to compare the accuracy of recognition. The algorithm is compared with Minitch stochastic gradient descent algorithm, and the results are shown in Table 4. Both algorithms have the worst recognition accuracy when SNR = 0.1 and the highest recognition accuracy when SNR = 0. However, under different SNR conditions, the recognition accuracy of the proposed algorithm is significantly higher than that of the Minitch stochastic gradient descent algorithm. indicating that the proposed classification algorithm can effectively improve the generalization ability of the model and the robustness of the model.

**Table 4:** Comparison of image recognition performance under different SNR.

SNR	0	0.03	0.05	0.07	0.1
The algorithm in the study	0.993	0.963	0.896	0.815	0.765
Minitch stochastic gradient descent algorithm	0.991	0.937	0.843	0.722	0.662

The results of this study are then compared with those of others. Eqs 7 and 8 are used to calculate the recall rate and accuracy of each algorithm.

$$P=\frac{TP}{TP+FP}$$ (7)

$$R=\frac{TP}{TP+FN}$$ (8)

Among them, P is the accuracy; R is the recall rate; TP is the true positive number; FP is false negative number; FN is the false positive number.

In this study, the recognition effect of the constructed network model is compared with SIFT [28], VGG19 [29], and Resnet [30]. The basic structures of SIFT, VGG19, and Resent network models are shown in Fig 9, Tables 5 and 6 respectively.

**Fig 9:** The basic structure of SIFT model.

**Table 5:** The basic structure of VGG19 model.

ConvNet Configuration					
A	A-LRN	B	C	D	E
11 weight layers	11 weight layers	13 weight layers	16 weight layers	16 weight layers	19 weight layers
Input (224*224 RGB image)					
Conv 3–64	Conv 3–64	Conv 3–64	Conv 3–64	Conv 3–64	Conv 3–64
	LRN	Conv 3–64	Conv 3–64	Conv 3–64	Conv 3–64
Maxpool					
Conv 3–128	Conv 3–128	Conv 3–128	Conv 3–128	Conv 3–128	Conv 3–128
		Conv 3–128	Conv 3–128	Conv 3–128	Conv 3–128
Maxpool					
Conv 3–256	Conv 3–256	Conv 3–256	Conv 3–256	Conv 3–256	Conv 3–256
Conv 3–256	Conv 3–256	Conv 3–256	Conv 3–256	Conv 3–256	Conv 3–256
			Conv 1–256	Conv 3–256	Conv 3–256
					Conv 3–256
Maxpool					
Conv 3–512	Conv 3–512	Conv 3–512	Conv 3–512	Conv 3–512	Conv 3–512
Conv 3–512	Conv 3–512	Conv 3–512	Conv 3–512	Conv 3–512	Conv 3–512
			Conv 1–512	Conv 3–512	Conv 3–512
					Conv 3–512
maxpool					
Conv 3–512	Conv 3–512	Conv 3–512	Conv 3–512	Conv 3–512	Conv 3–512
Conv 3–512	Conv 3–512	Conv 3–512	Conv 3–512	Conv 3–512	Conv 3–512
			Conv 1–512	Conv 3–512	Conv 3–512
					Conv 3–512
Maxpool					
FC-4096					
FC-4096					
FC-1000					
Soft-max					

The article "Analysis of the role and robustness of artificial intelligence in commodity image recognition under deep learning neural network" was retracted in 2024. Reasons: duplicate publication; overlap with earlier publications; compromised peer review; unreliable results or conclusions.

**Table 6:** The basic structure of Resnet model.

Layer-name	Output size	18-layer	34-layer	50-layer	101-layer	152-layer
Conv1	112*112	7*7, 64, stride 2				
Conv2_x	56*56	3*3 max pool, stride 2				
		$\left[\begin{array}{l} 3*3,64\\ 3*3,64 \end{array}\right]*2$	$\left[\begin{array}{l} 3*3,64\\ 3*3,64 \end{array}\right]*3$	$\left[\begin{array}{l} 1*1,64\\ 3*3,64\\ 1*1,256 \end{array}\right]*3$	$\left[\begin{array}{l} 1*1,64\\ 3*3,64\\ 1*1,256 \end{array}\right]*3$	$\left[\begin{array}{l} 1*1,64\\ 3*3,64\\ 1*1,256 \end{array}\right]*3$
Conv3_x	28*28	$\left[\begin{array}{l} 3*3,128\\ 3*3,128 \end{array}\right]*2$	$\left[\begin{array}{l} 3*3,128\\ 3*3,128 \end{array}\right]*4$	$\left[\begin{array}{l} 1*1,128\\ 3*3,128\\ 1*1,512 \end{array}\right]*4$	$\left[\begin{array}{l} 1*1,128\\ 3*3,128\\ 1*1,512 \end{array}\right]*4$	$\left[\begin{array}{l} 1*1,128\\ 3*3,128\\ 1*1,512 \end{array}\right]*8$
Conv4_x	14*14	$\left[\begin{array}{l} 3*3,256\\ 3*3,256 \end{array}\right]*2$	$\left[\begin{array}{l} 3*3,256\\ 3*3,256 \end{array}\right]*6$	$\left[\begin{array}{l} 1*1,256\\ 3*3,256\\ 1*1,1024 \end{array}\right]*6$	$\left[\begin{array}{l} 1*1,256\\ 3*3,256\\ 1*1,1024 \end{array}\right]*23$	$\left[\begin{array}{l} 1*1,256\\ 3*3,256\\ 1*1,1024 \end{array}\right]*36$
Conv5_x	7*7	$\left[\begin{array}{l} 3*3,512\\ 3*3,512 \end{array}\right]*2$	$\left[\begin{array}{l} 3*3,512\\ 3*3,512 \end{array}\right]*3$	$\left[\begin{array}{l} 1*1,512\\ 3*3,512\\ 1*1,2048 \end{array}\right]*3$	$\left[\begin{array}{l} 1*1,512\\ 3*3,512\\ 1*1,2048 \end{array}\right]*3$	$\left[\begin{array}{l} 1*1,512\\ 3*3,512\\ 1*1,2048 \end{array}\right]*3$
	1*1	Average pool, 1000-d fc, softmax				

At present, SIFT, VGG19, and Resnet are commonly used in image recognition. VGG19 contains 16 convolution layers (the size of convolution kernel is 3*3), 5 maximum pooling layers, and 3 fully connected layers. The activation function is ReLU. Resnet is also a classical structural model, and the activation function is ReLU. These two training methods, training data set, and iteration times are consistent with the MS-CNN model constructed in this study.

The article "Analysis of the role and robustness of artificial intelligence in commodity image recognition under deep learning neural network" was retracted in 2024. Reasons: duplicate publication; overlap with earlier publications; compromised peer review; unreliable results or conclusions.

It can be concluded from Table 7 that the recall rate and accuracy of the method constructed in this study are both greater than 90%. Moreover, the method constructed in this study can be used in the recognition and classification of single and multiple commodity images, and greatly improves the recognition performance. However, the recognition effect of VGG19 and Resnet model is poor. It may be because that from the recognition of a single commodity image to the recognition and positioning of multiple commodity images, the cross-task recognition makes the performance of the two models very low.

**Table 7:** Comparison of commodity recognition performance of different methods.

Methods	Recall rate	The accuracy
SIFT [28]	0.335	0.203
VGG19 [29]	0.365	0.263
Resnet [30]	0.587	0.429
The research method	0.929	0.971

## 5. Conclusion

In order to realize the automation and intelligent recognition of commodities, the commodity recognition platform is constructed based on the improved MS-CNN model. Then, the self-built commodity image database is used to train and verify the model. The results show that different convolution kernel sizes, Dropout rates, and label errors all affect the performance of image recognition, while the commodity image recognition method based on MS-CNN model in this study can effectively identify commodity images in complex scenes. However, the model constructed is only verified through self-built database, and not compared with other models. In the future, it is necessary to increase the sample size to explore the differences between the model constructed in this study and other models. To sum up, the establishment of the model in this study can lay a foundation for the realization of intelligent commodity recognition.

## Supporting information

S1 File (DOC)

S1 Data (XLS)
